# The forkhead-box family of transcription factors: key molecular players in colorectal cancer pathogenesis

**DOI:** 10.1186/s12943-019-0938-x

**Published:** 2019-01-08

**Authors:** Paul Laissue

**Affiliations:** Center For Research in Genetics and Genomics-CIGGUR, GENIUROS Research Group, School of Medicine and Health Sciences, Universidad del Rosario, Carrera 24 N° 63C-69, Bogotá, Colombia

**Keywords:** Colorectal cancer, Forkhead transcription factors, Molecular aetiology

## Abstract

Colorectal cancer (CRC) is the third most commonly occurring cancer worldwide and the fourth most frequent cause of death having an oncological origin. It has been found that transcription factors (TF) dysregulation, leading to the significant expression modifications of genes, is a widely distributed phenomenon regarding human malignant neoplasias. These changes are key determinants regarding tumour’s behaviour as they contribute to cell differentiation/proliferation, migration and metastasis, as well as resistance to chemotherapeutic agents. The forkhead box (FOX) transcription factor family consists of an evolutionarily conserved group of transcriptional regulators engaged in numerous functions during development and adult life. Their dysfunction has been associated with human diseases. Several *FOX* gene subgroup transcriptional disturbances, affecting numerous complex molecular cascades, have been linked to a wide range of cancer types highlighting their potential usefulness as molecular biomarkers. At least 14 *FOX* subgroups have been related to CRC pathogenesis, thereby underlining their role for diagnosis, prognosis and treatment purposes.

This manuscript aims to provide, for the first time, a comprehensive review of *FOX* genes’ roles during CRC pathogenesis. The molecular and functional characteristics of most relevant FOX molecules (FOXO, FOXM1, FOXP3) have been described within the context of CRC biology, including their usefulness regarding diagnosis and prognosis. Potential CRC therapeutics (including genome-editing approaches) involving *FOX* regulation have also been included. Taken together, the information provided here should enable a better understanding of *FOX* genes’ function in CRC pathogenesis for basic science researchers and clinicians.

## Background

Colorectal cancer (CRC) is a public health concern as it accounts for over 9% of all cancer incidence, representing > 1.4 million of new cases per year [1, 2]. It is the third most commonly occurring cancer worldwide and the fourth most frequent cause of death having an oncological origin [3]. Several risk factors have been related to CRC, such as inflammatory bowel disease, antecedents of CRC in first-degree relatives, increased body mass index, cigarette smoking, little physical activity and particular dietary habits [4]. Adenomas of the colon, which can be conventional adenomas or sessile serrated polyps, are the precursor lesions leading to most cases of CRC [5]. CRC has to be considered a complex disease resulting from a combination of environmental factors, genetic/epigenetic predisposing variants and specific molecular mechanisms. Three molecular pathways have been defined as major factors contributing to CRC carcinogenesis: microsatellite instability (MSI), chromosomal instability (CIN) and the CpG island methylator phenotype (CIMP) [6, 7].

The dysfunction of several genes in sporadic and familial cases has been associated with the disease’s aetiology, such as *KRAS*, *BRAF*, *c-Src*, *c-Myc*, *APC*, *TP53*, *PIK3CA*, *MSH2*, *MLH1*, *STK11*, *MSH6*, *PMS2*, *APC*, *CACNA1G*, *CDKN2A*, *IGF2*, *NEUROG1*, *RUNX3* and *SOCS1* [8, 9]. Some of these are currently used as clinically useful prognostic and therapeutic biomarkers [10]; indeed, since CRC development may take years, its early detection and the use of biochemical and molecular/genetic diagnostic tools is a keystone for improving survival rates.

The evolution of omics sciences’ experimental procedures during the last few years has led to new cancer classifications based on particular molecular findings underlying tumour’s biology [11–13]. For instance, immune-MSI, canonical-CMS2, metabolic-CMS3 and mesenchymal-CMS4 CRC subtypes have been proposed based on transcriptomic differences between tumours which should improve the disease’s diagnosis/prognosis/treatment. Interestingly, it has been found that transcription factor (TF) dysregulation, mainly due to chromosomal deletion/translocation/amplification and point mutations, is a widely distributed phenomenon regarding human malignant neoplasias [14–16]. TF dysregulation can lead to the significant expression modifications of genes involved in various complex biological processes, such as cell identity determination, proliferation regulation and cell signalling for controlling machinery in response to micro-environmental signals [17]. These changes are key determinants regarding tumour’s behaviour as they contribute to cell differentiation/proliferation, migration and metastasis, as well as resistance to chemotherapeutic agents.

Since the first association was made between DNA regulatory regions and phenotypic variation in bacteria, considerable efforts and advances have been made to understand TFs’ genomic regulation, such as reporting new gene families, identifying genetic and epigenetic molecular modulatory mechanisms, describing expression profiles and programmes regarding numerous cell types, studying the evolution of genetic networks, developing omics data analysis and characterising variations on regulatory motifs and TF mutations in human disease-related encoding regions [15, 18–31]. TFs have been classically organised into families and subfamilies, depending on the sequence/structure of their DNA binding domain (DBD) [29]. The total amount of TFs has not yet been precisely stated; however, at least 1400 have high confidence sequence-specific DBD [20]. Mechanistically TFs recognise 6–12 bp-long DNA sequences located on target gene promoters/enhancers to regulate expression. These motifs, known as transcription factor binding sites (TFBS), provide specificity for binding and their occupancy has been related to several variables such as quantity, affinity and availability of regulatory complexes in specific regions [28, 32]. TFs bind to other proteins (e.g. cofactors) to form macromolecular complexes which are essential elements for specific binding to TFBS and establishing complex regulatory networks [33–35].

The forkhead box (FOX) transcription factor family consists of an evolutionarily conserved group of transcriptional regulators engaged in numerous functions during development and adult life; their dysfunction has been associated with human diseases [36–42]. Several *FOX* gene subgroup transcriptional disturbances, affecting numerous complex molecular cascades, have been linked to a wide range of cancer types highlighting their potential usefulness as molecular biomarkers [23, 41–49]. At least 14 *FOX* subgroups have been related to CRC pathogenesis, thereby underlining their role for diagnosis, prognosis and treatment purposes.

This manuscript aims to provide, for the first time, a comprehensive review of *FOX* genes’ roles during CRC pathogenesis. The molecular and functional characteristics of most relevant FOX molecules have been described within the context of CRC biology, including their usefulness regarding diagnosis and prognosis. Potential CRC therapeutics (including genome-editing approaches) involving *FOX* regulation have also been included. Taken together, the information provided here should enable a better understanding of *FOX* genes’ function in CRC pathogenesis for basic science researchers and clinicians.

## Main text

### The FOX family of transcription factors: an overview

The first report of a *FOX* gene was published in the late 1980s when a mutant model of *Drosophila melanogaster* was described as having a transformation of the foregut resembling a head-like structure [50, 51]. Since then, at least 50 additional members, which have been classified in 19 subgroups (FOXA to FOXS), have been discovered in human species [37, 40, 52–54]. All FOX members share a highly conserved ~ 100 residue DBD (the forkhead domain, FOX-DBD) which was first identified in *Drosophila* forkhead and mammalian HNF-3a (FOXA1), HNF-3b (FOXA2), HNF-3c (FOXA3) proteins [50, 52, 55]. The FOX-DBD binds to a target genes’ core sequence (5′-(G/A)(T/C)(A/C)AA(C/T)A-3′) located on the promoter regions [38]. Sequences adjacent to the core TFBS are also important for TF differential affinity and functions [56–58]. Structurally, the FOX-DBD consists of three N-ter α-helices, three β-strands and two loops, resembling butterfly wings or a “winged helix” [38, 59, 60]. However, some FOX-DBD have some modifications in their secondary structure composition and topological arrangements [60] (and references therein). It has been shown that the wings contribute to regulating DNA binding specificity and affinity [61].

Several post-translational modifications, such as phosphorylation, acetylation and ubiquitination, have been described which contribute to modulating different FOX proteins’ functions, including their DNA-binding affinity [60]. Functional regions in addition to the DBD have been mapped for some FOX proteins, such as the FOXO subfamily, i.e. the transactivation domain (TAD), the nuclear localisation sequence (NLS) and the nuclear export sequence (NES) (Fig. 1). Contrary to the DBD, such regions are poorly conserved and may contain variable length homopolymeric tracts (e.g. Ala, Gln, Pro residues). In some cases (FOXL2, FOXP2) these regions´ length can be modified above/below a threshold leading to cellular dysfunctions contributing to causing the disease [62–64]. To date, the Protein Data Bank-DBD contains the structure of the FOX-DBD bound to the DNA of several FOX members: FOXA1, FOXA2, FOXM1, FOXN1, FOXO1, FOXO2, FOXO4, FOXK1, FOXK2, FOXP1, FOXP2 and FOXP3 [65] (https://www.rcsb.org/).

**Fig. 1:** Structure of FOXO3A, FOXM1 and FOXP3 proteins. DBD: DNA binding domain (forkhead domain); NLS: nuclear localisation sequence; NES: nuclear export sequence; TAD: transactivation domain; NRD: negative-regulatory domain; TRD: transcriptional repressor domain; LZ: leucine zipper motif

FOX proteins are widely distributed throughout multiple species from yeasts to humans and play pleiotropic roles in developmental and adult age biological/cellular processes, such as cell cycle control, cell differentiation and proliferation, tissue homeostasis, aging, metabolism regulation and stress tolerance. FOX factors are key regulators of various signalling pathways regarding physiological and pathological conditions: phosphatidylinositol 3-kinase/protein kinase B (PI3K-AKT), transforming growth factor beta (TGF-β), WNT/β-catenin, insulin, Sonic-Hedgehog and Jagged-Notch [38] (and references therein). *FOX* gene deregulation in cancer pathophysiology brings consequences regarding its onset, maintenance, progression and drug resistance. FOX molecules constitute therefore molecular biomarkers for diagnostic and prognostic purposes. Furthermore, they form coherent potential targets for therapeutic approaches, including genome editing-based strategies.

### A dual role for FOXOs as tumour suppressors and potential oncogenic proteins

The FOXO subfamily of forkhead transcription factors, which has been widely studied during last 20 years, consists of four members in mammals: FOXO1, FOXO3A, FOXO4 and FOXO6. Structurally, these proteins include the forkhead (FKH) and TAD domains and nuclear localisation and exports signals [42, 66] (Fig. 1). All FOXO proteins have high FKH domain homology, particularly in the N-ter region (RXRSCTWPL motif) [40]. Concerning target DNA regions, FOXO proteins recognise the Daf-16 family member binding element (5′-GTAAA(T/C)AA-3′) and the insulin-responsive element (5′-(C/A)(A/C)AAA(C/T)AA-3′) for regulating gene expression [67]. FOXO molecules are expressed in numerous tissues during embryo development and adult life, and have been related to different functions such as cell differentiation/proliferation, controlling metabolism, immunity, apoptosis, detoxification, DNA damage repair, cell cycle arrest, autophagy, homeostasis maintenance, modulating stress resistance and aging [39, 42, 68–76].

Upstream regulation of FOXO subfamily members has been well documented, especially the mechanism involving the phosphoinositide-3-kinase–protein kinase B (AKT) (PI3K-AKT) molecular cascade in response to insulin and growth factor stimulation [69, 77] FOXOs phosphorylation by AKT (on Thr^32^, Ser^253^ and Ser^315^ residues) enables its binding to 14-3-3 proteins; the complex so formed is then translocated from the nucleus to the cytoplasm [78] (Fig. 2). In addition to AKT, other kinases (e.g. SGK, IKK, ERK) are negative regulators of FOXO, while JNK and MST1 are able to activate it [79, 80].

Regarding cancer biology, FOXO proteins acts downstream of several oncogenic pathways such as, PI3K–AKT, ERK and NF-κB-IKKβ (nuclear factor-κB and NF-κB kinase-β inhibitor, respectively) [39, 77, 81–83]. FOXOs have mostly been described as tumour suppressors as they possess anti-proliferative and pro-apoptotic properties. FOXOs’ anti-tumour function has been related to the regulation of key genes participating in cell death and cell cycle arrest, such as *p27*^*KIP1*^, *CDKN1A/p21*, *FasL*, *Trail* and *Bim* [80, 84, 85]. FOXOs are also involved in other complex networks, including numerous genes regulating the relevant process of tumorigenesis, such as oncogene-induced senescence, angiogenesis, invasiveness, oxidative stress regulation and interaction with other suppressors (e.g. p53).

A dual yet paradoxical role has been described for *FOXO* in CRC, as they can act as a cancer suppressor genes or an oncogenes (see below). It has been shown, in colon carcinoma-derived cells, that the FOXO system activation/inhibition via gene overexpression/silencing or the pharmacological perturbation of several signalling pathways (PI3K-AKT, Wnt, β-catenin, EGFR) lead to CRC cancerogenesis [86–115].

Numerous studies have described FOXO participation in regulating the PI3K/AKT molecular cascade, a signalling pathway which becomes altered in most human cancers (Fig. 2). The PI3K is a family of lipid kinases involved in several key cellular processes such as differentiation, proliferation/growth, survival, metabolism and migration [116] (and references therein). This pathway is associated with different nodes constituted by numerous molecules, underlining different functions and having particular regulatory complexity. The PI3K pathway can be activated by different types of signal, including receptor tyrosine kinases (RTKs) and G-protein-coupled receptors and oncogenes leading to plasma membrane recruitment and the activation of class I PI3K family proteins [117]. PI3K activity enables AKT membrane recruitment; thereafter, AKT becomes activated, in turn, leading to the phosphorylation of different effectors, such as FOXOs, GSK3, eNOS, TSC2, BAD and p27. It has been shown that AKT activation induces FOXO3 accumulation in the cytoplasm via 14-3-3 protein action, thereby inhibiting its function [81, 118] (Fig. 2).

**Fig. 2:** Regulation of FOXO subcellular distribution and activity via PI3K/AKT activation. In the presence of growth factors the PI3K/AKT system is activated and the FOXO-TFs are phosphorylated. This modification creates a docking site for 14–3-3, which excludes FOXOs from the nucleus inhibiting the transactivation of target gene promoters (red arrow). In the contrary, the absence of growth factors and AKT/PI3K activation allows FOXO nuclear translocation and the transactivation of target gene promoters (green arrow). GF: growth factors

Several reports have studied the effect of FOXO activation/inactivation on CRC biology. Ericson et al. [111] used target homologous recombination in CRC cells to inactivate the *AKT1*, *AKT2* or *PDPK1* genes. The Akt1/Akt2 double KO, which was related to a substantial decrease in FOXO1A and FOXO3A phosphorylation, led to considerably reduced cell proliferation in vitro and perturbed metastasis in mice. The results suggested that the expression of genes, secondary to phosphorylated FOXO proteins’ decreased activity in the nucleus, contributed to AKT factors’ growth-promoting function. This effect appeared to be independent of other important PI3K signalling pathway molecules, such as mammalian target of rapamycin (mTOR) and glycogen synthase kinase 3 beta (GSK3β).

Depletion of the PI3K regulatory subunit p85α via siRNA transfection in LoVo and SW480 colorectal cell lines inhibited cell proliferation, induced G1 phase cell cycle arrest and sensitised colorectal cancer cells to 5-FU-induced apoptosis [112]. The lack of p85α in these experiments led to a strong decrease in AKT (and phosphorylated AKT) which led to a significant decrease of FOXO proteins (FOXO1, FOXO3A and FOXO4) in the cytoplasmic compartment. A logical accumulation of these factors was observed in the nucleus which was related to some target genes’ expression modification (e.g. cyclin D1 and cdk4 were downregulated while p27/Kip1 and FasL were upregulated). Seminal work by Tenbaum et al., studied the crosstalk between WNT–β-catenin and PI3K-AKT-FOXO3A pathways in CRC tumorigenesis [115]. The authors explored the simultaneous effect of WNT–β-catenin molecule hyper-activation and PI3K-AKT inhibition on CRC biology. This scenario was related to FOXO3A and β-catenin nuclear accumulation, in turn, being related to a cell scattering phenotype and metastasis. It has been defined that FOXO3A and β-catenin regulate many metastasis-relevant genes, such as *IQGAP2*, *CYR61*, *CLDN1*, *CAV1*, *EDN1* and *KIT*. Indeed, various metastasis-related biological processes are modulated (via target genes) by FOXO3A and β-catenin, such as cell motility and migration, angiogenesis, immune system evasion and cytoskeleton reorganisation. Nuclear β-catenin resistance to FOXO3A-mediated apoptosis has been induced by PI3K and AKT inhibitors in primary CRC cells. Interestingly, high FOXO3A and β-catenin nuclear concentrations have been related to the CRC metastatic stage and affected patients’ shorter survival times [115]. Contrary to that reported by others, these findings add information regarding FOXO3A’s potential oncogenic nature.

Shoeb et al. [90] have shown that aldose reductase inhibition, via PI3K/AKT, modulated FOXO3A activation in CRC cells, in turn, participating in sensitising tumour cells to tumour necrosis factor –TNF-related apoptosis-inducing ligand (TRAIL)-induced apoptosis. Several other studies have described the effect of FOXO accumulation in the nucleus of CRC cells, some of which were based on using different kinds of molecules. For instance, cisplatin was administered to various CRC cell lines to assess the role of the PI3K/FOXO pathway in such drug action and resistance [109]. Cisplatin caused apoptosis in sensitive cells and modified long-term cell survival, which was linked to FOXO3A nuclear translocation. FOXO3A dephosphorylation became impaired in resistant cells, thereby affecting target gene promoter transactivation (i.e. p27Kip1 and BIM). Cisplatin use, combined with p38α pharmacological inhibition, has also been shown to be related to decreased cancer cell viability through increasing BAX-dependent apoptotic cell death by activating FOXO3A tumour suppressor properties [92]. Such activation was related to p21, *PTEN*, *BIM* and *GADD* upregulation, inducing apoptosis in CRC cells.

In another study, Luo et al., demonstrated that treating HCT116 and SW480 CRC cells with selenite inhibited AKT and the consequent accumulation of FOXO3A, thereby facilitating the transcription of target genes such as *BIM* and *PTEN* [88]. FOXO3A-mediated upregulation of PTEN contributed to enhancing the inhibitory effect on the AKT pathway. Selenite therefore seemed to induce ROS-dependent FOXO3A-mediated apoptosis in CRC cells. Regarding inflammation, treating HCT-8 and HCT116 cells with docosahexaenoic acid (DHA, an omega-3 polyunsaturated fatty acid) produced the nuclear accumulation of FOXO3A, which bound to the miR-21 promoter, activating its repression [101]. The study by Fluckiger et al., demonstrated that RIP1 and AMPKα regulated FOXO3A-miR-21 signalling, modulating TNFα production after DHA treatment of CRC cells; this approach led to tumour growth inhibition and apoptosis. Administering genistein, a prominent component of soy, inhibited EFG-induced proliferation in HT-29 cells, favouring FOXO3A nuclear retention [86]. Other studies have described similar results when using other treatments such as cetuximab (a monoclonal antibody against EGFR) and quinazoline [95, 103].

Regarding studies describing reduced FOXO nuclear bioavailability, experimental approaches have included genetic engineering of cells and animal models, drug treatment and gene expression knock-down. It has been shown that proliferation of colonic epithelia and CRC cells via EGFR stimulation has been associated with a loss of FOXO3A activity (phosphorylation, translocation to the cytosol and degradation) and a decrease in its transactivation properties regarding the *p27kip* promoter [87]. Dehner et al., studied the transcriptional effect of WNT signalling pathway over-activation on HCT-116 cells [110]; they found that the *SGK1* gene was the most up regulated gene, thereafter leading to FOXO3A nuclear exclusion. This change in protein bioavailability in the nuclear compartment was associated with the inhibition of target gene expression and FOXO3A-induced apoptosis.

Another interesting study described the stimulation of intracytoplasmic lipid droplet (a dynamic organelle present in tumour tissues) density in human colon cancer cells which led to the loss of FOXO3A (via PI3KB) and a decrease in Sirtuin6 (SIRT6) lipid metabolism [89]. Furthermore, dissociation of FOXO3A from the *p27kip1* promoter (and its subsequent decreased expression) stimulated CRC cell proliferation; a negative regulatory loop between LDs and FOXO3/SIRT6 was identified thereafter [99].

It has been shown that the DEAD box protein P68 (p68) and FOXO3A have differential expression in CRC (up- and down-regulation, respectively) [97]. Indeed, p68 has been seen to be related to a reduction in FOXO3A, via AKT, which contributed to CRC oncogenesis in vitro and in vivo. Similarly, high REP1 (Rab escort protein) expression has been linked to a direct blockade (REP1 and FOXO3A are direct protein partners) of FOXO3A nuclear trans-localisation in CRC cells, which has suppressed FOXO3-mediated apoptosis [104]. In that study, REP1 inhibition, combined with 5-FU treatment, led to retarding tumour growth in mice, leading to it being proposed as a potential therapeutic target for CRC. FOXO3A inactivation has been related to reactive oxygen species (ROS) production during protein kinase CK2 downregulation-mediated senescence in human CRC cells [102]. This effect was facilitated by AKT-mediated phosphorylation of FOXO3A and the decreased transcription of several target genes, such as Cu/ZnSOD, MnSOD and catalase (CAT). Using Nlrc3^−/−^ mice has enabled showing that Nlrc3 regulates cell proliferation in CRC by reducing FOXO3A and FOXO1 activation [105, 119]. These findings argue in favour of the therapeutic potential of regulating NLRC3 for treating CRC.

More recently it has been shown that Rho GTPase-activating protein 15 (RHGAP15) and FOXO1 expression was lower in CRC specimens than in normal colonic mucosa [106]. An increase in PTEN and FOXO1 was observed in ARHGAP15-overexpressed HT29 and RKO cells, along with decreased AKT phosphorylation. It was concluded that PTEN/AKT/FOXO1 signalling was participating in ARHGAP15 anti-proliferation and anti-invasion effects.

A series of studies has shown that *FOXO* transcript expression knock-down has enabled understanding potential regulatory mechanisms involved in CRC pathogenesis; indeed, different microRNAs (miRNA) have been studied in vivo and in vitro to assess FOXO tumour suppressor properties. It has been shown that miR-544 binds FOXO1, while miR-153 and miR-592 bind FOXO3A [91, 100, 120]. miR-96 has been described as binding to both FOXO1 and FOXO3A [94]. In all these cases the molecules’ effects have contributed to CRC biology.

Most histopathological reports aiming to associate FOXO expression/localisation with disease outcome in cancer patients have described a role for FOXOs as tumour suppressors. Studying primary CRC tissues and their corresponding metastases has shown that FOXO3A levels became decreased during metastasis, thereby evoking a role for this protein as a cancer suppressor [45, 76]. However, its nuclear localisation has also been linked to lower overall CRC survival [115]. Taken together, these results pinpoint the complexity of FOXO regulatory networks and reinforce these transcription factors’ dual role as cancer suppressors and oncogenes. In this context, using FOXOs expression levels for CRC diagnostic/prognostic purposes remains limited. Indeed, transcriptional data from CRC should be analysed globally considering dysregulation of key biological processes and molecular pathways. Interestingly, Tenbaum et al. have proposed the measurement of nuclear β-catenin as a biomarker of treatments leading to FOXO3A nuclear accumulation, which might predict apoptosis or metastasis [115]. In addition, this may be useful for molecules acting upstream, as AKT/PI3K and tyrosine kinase inhibitors.

### FOXM1: a major actor in cell cycle regulation

The *FOXM1* gene (also known as *MPP-2*, *WIN*, *HFH-11* and *Trident*), which is located at 12p13–3 in human species, has 10 alternatively spliced exons, leading to the synthesis of 3 protein isoforms (FOXM1a, b and c) [43, 121, 122]. It has been reported that the FOXM1 DBD was able to bind the canonical FKH motif (5′-RYAAAYA-3′) on DNA for regulating target genes. Structurally, FOXM1 has several functional domains: the DBD, a strong acidic TAD located in the protein’s C-terminal region, and a negative-regulatory domain in the N-terminal (NRD) [39] (and references therein) (Fig. 1). FOXM1 is well known for its function during cell cycle regulation and its localisation in the nuclear compartment depends on ERK phosphorylation on Ser^331^ and Ser^704^ residues [123]. It has been shown that the impaired activation of several receptor tyrosine kinases, such as RTK, RAF, RAS and MAPK2, in cancer cells has led to the nuclear accumulation of FOXM1, via ERK phosphorylation. FOXM1 is a master factor involved in G1/S and G2/M cell cycle transition and M phase progression. It has been linked to normal chromosomal stability and segregation during mitosis [43]. FOXM1 has been associated with cellular senescence, stem cell-like self-renewal, cell differentiation and proliferation, tissue homeostasis, cell migration and invasion, DNA damage repair and angiogenesis, oxidative stress regulation, and drug resistance during tumorigenesis.

Regarding CRC biology, FOXM1 expression levels have been reported to be correlated with cancer progression, lymph node and liver metastasis and high TNM stages [124–127]. These findings agreed with decreased patient survival rate. Interestingly, high concurrent FOXM1 and CAV-1 (caveolin 1) overexpression plays an important role in CRC development and progression by negatively regulating E-cadherin [128].

The hedgehog (Hh) signalling and the GLI proteins have been shown to be important actors in CRC development. *Hh* genes encode secreted proteins functioning as intercellular signalling molecules and participating in several developmental and adult tissue biological processes. GLI are zinc finger transcription factors, mainly having activating properties regarding target genes including *Hh*, some of which (e.g. GLI1) have proto-oncogenic properties. Douard et al., found that overexpression of *Sonic Hedgehog*-*SHh*- (a member of the Hh family), *GLI1* and *FOXM1* was linked to increased cell proliferation in primary CRC tissue and cell lines [129]. It has recently been proven that GLI1 directly binds to and transactivates the FOXM1 promoter [130, 131] (Fig. 3). GANT61-treated HT-29 cells have displayed FOXM1 transcriptional impairment secondary to the inhibition of GLI binding to chromatin and RNA polymerase to DNA [132]. Interestingly, GLI also participates in CRC metastasis by activating (via FOXM1) EMT and PI3K/AKT signalling pathways [131]. Regarding target gene downstream regulation, FOXM1 directly binds to PTTG1 and HSPA5 promoters participating in CRC cell invasion and migration [133, 134] (Fig. 3). Furthermore, FOXM1 directly binds to and transactivates the growth arrest–specific (GAS1) promoter of a gene involved in the negative regulation of oncogenesis and CRC metastasis [135, 136]. The Fig. 3 includes a comprehensive list of regulators of FOXM1 and its effector genes.

**Fig. 3:** FOXM1 upstream regulators and downstream effectors

Interestingly, FOXM1 has also been described as a relevant actor during mitochondrial metabolism. For instance, FOXM1 expression has activated peroxiredoxin-3 (Prx3) mitochondrial gene transcription and CD133 expression in colon cancer stem cells (CSC) [137, 138]. Increased *PRX3* expression by FOXM1 has been seen to be related to mitochondrial activity maintenance via the elimination of ROS, thereby leading to colon CSC survival and stemness. A novel FOXM1 isoform has been identified more recently: FOXM1D [139]; FOXM1D has an essential function in Rho/ROCK activation, a signalling pathway involved in actin cytoskeleton organisation and cancer invasion. More precisely, FOXM1D overexpression contributes to actin assembly polymerisation and interferes with E-cadherin expression, which is related to metastasis.

Regarding miRNA mechanisms leading to FOXM1 knock-down, it has been shown that the downregulation of miR-320, miR-149, mi-R-342 is related to CRC biology [140–144]. Notably, miR-320 and miR-342 are suppressors of both FOXM1 and FOXQ1, constituting potentially interesting therapeutic tools for CRC [143, 144]. Clinically, FOXM1 may be used directly as a diagnostic/prognostic marker as high expression levels have been correlated, in independent cohorts of CRC patients, with poor survival [144]. In addition, due to its clear oncogenic nature FOXM1 has emerged as promissory target for cancer drug therapy [145].

### FOXP3: a molecule at the crossroads of immunity and tumorigenesis

The long story of the *FOXP3* gene goes back 50 years to when the Oak Ridge National Laboratory’s Mammalian Genetics Laboratory (USA) explored the genetic consequences of radiation on mammals [146]. This initiative led to the description of one of the most well-known strains of mouse having a spontaneous mutation carried by the X chromosome: the “scurfy” mouse [147, 148]. It was stated that these animals’ phenotype (characterised by scaly and ruffled skin, reddened eyes, abnormal spleen and lymph node growth and early death) originated from a *Foxp3* 2 bp out-of-frame insertion leading to a truncated protein product. Functionally, the phenotype was associated with an autoimmune phenomenon and a suppressor T-cell subset expressing *Foxp3*, CD4 and CD25 [149]. Thereafter, *Foxp3* was described as a major molecular actor involved in regulatory T-cell (Treg) development and function [150–152]. The loss of *Foxp3* in mice leads to a fatal lymphoproliferative disorder whilst its overexpression causes an immunodeficiency phenotype [153, 154]. *FOXP3* germline mutations in humans have been associated with the X-linked autoimmunity-allergic dysregulation syndrome, also known as immunodysregulation, polyendocrinopathy and enteropathy, X-linked (IPEX) syndrome [155–157].

*FOXP3* is located in Xp11.23 in human beings and has 11 encoding exons which are translated into a 431-residue (47 kDa)-long protein [155]. Structurally, from the N-ter to the C-ter regions, FOXP3 consists of a proline-rich transcriptional repressor domain (TRD), a zinc finger, a leucine zipper motif (LZ) and the FOX-DBD containing the NLS [39, 158] (Fig. 1). Two principal FOXP3 isoforms are synthesised in human species, one issuing from the translation of the full length open reading frame and another lacking a specific region involved in retinoic acid-related orphan receptor (RORα) inhibition [159]. *FOXP3* is mainly expressed by Treg cells, but it has also been found in other cells (e.g. B-lymphocytes) and various normal tissues (e.g. breast, prostate, lung, thymus, colon, kidney, ovary) [154, 160–162].

Interestingly, it has been found that Treg cells infiltrate various types of tumour-related tissue in mouse and human species, such as lung, liver, breast, ovary, pancreas, head, neck, gastrointestinal tract, skin and other tissues [163–165] (and references therein). The discovery of somatic mutations and epigenetic alterations has revealed a dual role for *FOXP3* regarding cancer biology as it can act as an oncogene or a tumour suppressor gene (e.g. breast, cancer and prostate) [162, 166–169]. Numerous human cancer cell lines, including some having a colorectal origin (e.g. HCA 2.6, HCA 3.2), have different *FOXP3* expression levels which has enabled assessing its function in different in vitro conditions [170]. Non-encoding sequence regulatory regions, minimal promoter trans-regulation and epigenetic mechanisms have been described regarding *FOXP3*’s upstream regulation [148].

Due to the close relationship between Treg cells and tumours’ microenvironment, *FOXP3* has been widely studied in CRC development and progression. At least 80 studies on FOXP3 and CRC biology have been published to date; however, the usefulness of FoxP3^+^-Tregs cells for clinical prognosis regarding CRC has been a subject for continuous debate. Xu et al., published a meta-analysis based on 18 previously-reported studies which examined > 3500 patients, aiming to determine FoxP3^+^ prognostic role in CRC [171]. Numerous variables were considered for analysis in that study, such as specimen type (e.g. tissue, tissue microarray, blood), *FoxP3*^*+*^ and other marker’s testing methods (e.g. immunohistochemistry-IHC, quantitative real time polymerase chain reaction (qRT-PCR), flow cytometry analysis (FCM), CRC tumour stage, follow up time and survival. It was found that high FoxP3^+^-Treg infiltration was linked to an improvement in cancer-specific survival. These findings were similar to those reported by Huang et al.’s meta-analysis (2014), but differed from those from other studies, probably due to differences in sample type and consistency during data analysis [171–177]. It has been shown that FoxP3^+^ non-T_reg_ cells can infiltrate some colorectal cancers (e.g. those having TGF-β and IL-12 expression) leading to a better prognosis. It is worth noting that the difficulty of separating cell subpopulations may be a relevant factor contributing to contradictory findings in research involving immunohistochemistry [163, 178].

Regarding *FOXP3*’s regulation, it has been shown that various proteins (e.g. NFAT, AP-1, FOXO1, FOXO3, CREB-ATF1, SAMD3, RAR-RXR, RUNX, ETS1, STAT5) are capable of directly binding to its promoter and other regulatory regions to activate its transcription [179–181]. The TGFβ molecule has been shown to be capable of inducing FoxP3 expression in CD4^+^CD25^+^ cells [160].

Regarding downstream regulation, it has been proposed that FOXP3 may bind to more than 2800 TFBS in T_reg_ cells, representing > 700 genes [182]; however, thousands of other genes are predicted to be indirectly regulated by FOXP3 via its interaction with numerous cofactors (e.g. NFAT, IRF4, RUNX1, EOS, IRF4, SATB1, LEF1, GATA1, TIP60 and p300) forming large protein complexes [181, 183, 184].

Thus, it can state that although the role of FOXP3 in CRC biogenesis is still not completely understood, numerous reports have argued in favour of a FoxP3+ Treg cell protective function by controlling carcinogenesis, improving local inflammation and, *in fine*, ameliorating patients’ chances of survival.

### Other FOX proteins involved in CRC biology

Several other FOX proteins have been described as important regulators of CRC tumorigenesis. However, since they have not been studied as extensively as those described above, they will not be widely reviewed in the present manuscript. For instance, FOXC1 and FOXC2 promote CRC metastasis by regulating *ITGA7*/*FGFR4* and *MET* expression, respectively [185–187]. It has been stated that FOXQ1 plays a key regulatory role in epithelial-mesenchymal transition of several types of cancer, including CRC [188, 189]. *FOXQ1* overexpression has been seen to play a relevant role in enhancing CRC tumorigenicity, tumour growth and migration/invasion of tumour cells by mainly acting on WNT and TGF-B molecular pathways [144, 190–192]. Other FOX proteins having oncogenic properties in CRC would include FOXA1, FOXD1, FOXD3, FOXF1, FOXF2 FOXJ1, FOXK1, FOXK2, FOXN3 and FOXR2 [46, 47, 65, 193–204]. Additional FOX TF studies have reported tumour suppressor properties for some of them, such as FOXE1, FOXF1, FOXF2 and FOXJ3 [205–210].

Although these factors deserve additional functional studies, some of them might be used in the future as diagnostic/prognostic studies for CRC.

### Targeting FOX molecules for CRC therapeutics and future research

As stated above, TFs can have oncogenic or tumour suppressor properties, acting on various key molecular cascades involved in CRC pathogenesis. Classically, except for ligand-inducible nuclear receptors, TFs have been described as “undruggable” targets. However, several recent approaches aiming to regulate TF activity (enhancing or inhibiting it) have been proposed, several of which have been used in cancer biology studies [16, 211–214]. Regarding suppressor TFs, increasing their function has been obtained by using pharmacological approaches while other chemical strategies have been used to restore their function. TF oncogenic function has been inhibited by targeting their cofactors in different ways, such as using small-molecule and short-based peptide based approaches. On the whole, targeting TF methods includes those aiming to regulate their expression/degradation, perturb their protein/protein interactions and act on the TFBS-DBD. FOX factors have not been widely explored using these strategies, thereby underlining an interesting field for potential research regarding CRC therapy. Recently, FOX factors have been studied concerning various biological processes using different experimental designs based on using the CRISPR/Cas9 genome editing tool [215, 216]. Future therapy will combine CRISPR/Cas9 specific genome editing with classic drug treatment; using this approach for modulating *FOX* gene function will certainly provide attractive therapy for CRC treatment.

## Conclusions

FOX TFs are key molecular actors during CRC, which can act in distinct molecular cascades regulating several biological processes. Their target regulation by using classical therapeutic approaches and/or novel techniques might improve CRC prognosis. Future research and treatment should therefore involve their study at genomic, transcriptomic and proteomic levels. Certainly, blocking FOX TFs oncogenic properties during CRC development will contribute to improve patient outcomes.

## Abbreviations

CIMP: CpG island methylator phenotype
CIN: Chromosomal instability
CRC: Colorectal cancer
DBD: DNA binding domain
FKH: Forkhead
FOX: The forkhead box
FOX-DBD: Forkhead domain
MSI: Microsatellite instability
NES: Nuclear export sequence
NLS: Nuclear localisation sequence
NRD: Negative-regulatory domain
TAD: Transactivation
TAD: Transactivation domain
TF: Transcription factors
TFBS: Transcription factor binding sites
